The article "Segmentation of Oral Leukoplakia (OL) and Proliferative Verrucous Leukoplakia (PVL) Using Artificial Intelligence Techniques" was retracted in 2023. Reasons: signs of a paper mill; suspected computer-generated content; unreliable results or conclusions; lack of ethics approval or compliance.

# Segmentation of Oral Leukoplakia (OL) and Proliferative Verrucous Leukoplakia (PVL) Using Artificial Intelligence Techniques

**DOI:** 10.1155/2022/2363410

**Published:** 2022-07-21

**Authors:** Samar Zuhair Alshawwa, Asmaa Saleh, Malek Hasan, Mohd Asif Shah

**Affiliations:** ^1^Department of Pharmaceutical Sciences, College of Pharmacy, Princess Nourah bint Abdulrahman University, P.O. Box 84428, Riyadh 11671, Saudi Arabia; ^2^Department of Medical Instruments Engineering Techniques, Al-Farahidi University, Baghdad 10021, Iraq; ^3^The University of Mashreq, Research Center, Baghdad, Iraq; ^4^Kebri Dehar University, Ethiopia

## Abstract

PVL (proliferative verrucous leukoplakia) has distinct clinical characteristics. They have a proclivity for multifocality, a high recurrence rate after treatment, and malignant transformation, and they can progress to verrucous or squamous cell carcinoma. AI can aid in the diagnosis and prognosis of cancers and other diseases. Computational algorithms can spot tissue changes that a pathologist might overlook. This method is only used in a few studies to diagnose LB and PVL. To see if their cellular nuclei differed and if this cellular compartment could classify them, researchers used a computational system and a polynomial classifier to compare OLs and PVLs. 161 OL and 3 PVL specimens in the lab were grown, photographed, and used for training and computation. Exam orders revealed patients' sociodemographics and clinical pathologies. The nucleus was segmented using Mask R-CNN, and LB and PVL were classified using a polynomial classifier based on nucleus area, perimeter, eccentricity, orientation, solidity, entropies, and Moran Index (a measure of disorderliness). The majority of OL patients were male smokers; most PVL patients were female, with a third having malignant transformation. The neural network correctly identified cell nuclei 92.95% of the time. Except for solidity, 11 of the 13 nuclear characteristics compared between the PVL and the LB showed significant differences. The 97.6% under the curve of the polynomial classifier was used to classify the two lesions. These results demonstrate that computational methods can aid in diagnosing these two lesions.

## 1. Introduction

According to the World Health Organization, cancer arises from transforming normal cells into tumor cells in a multistage process [1]. Among the various types of tumors, squamous cell carcinoma (SCC) of the oral cavity is usually preceded by MPDs, which develop from etiological factors such as tobacco, alcohol, autoimmune diseases, and idiopathic or inherited genetic aberrations. We can mention oral leukoplakia (OL), erythroplakia, oral submucosal fibrosis, palatine keratosis associated with inverted smoke, lichen planus, lupus erythematosus, and dyskeratosis congenita [2]. Although each of them has specific histological aspects, some histological characteristics such as hyperkeratosis (increase in keratin), hyperplasia (increase in the number of cells), and even dysplasia (an architectural disorder of epithelial tissue accompanied by cytological atypia) may be shared between them [3].

The article "Segmentation of Oral Leukoplakia (OL) and Proliferative Verrucous Leukoplakia (PVL) Using Artificial Intelligence Techniques" was retracted in 2023. Reasons: signs of a paper mill; suspected computer-generated content; unreliable results or conclusions; lack of ethics approval or compliance.

Premalignant cases are local lesions characterized by a higher risk of malignant change than normal structures or general conditions associated with an increased risk of cancer. Oral mucosa is an area where more than 5% of premalignant cases turn into cancer [4, 5]. Therefore, the diagnosis of premalignant formations gains importance in the early detection of possible malignant lesions. Problems in evaluating premalignant cases mainly arise from two factors [5]. Although various clinical features are important in determining the risk of malignant change in premalignant cases, histological examinations are the most valid method today to determine these formations' proper structure and malignant potential. Histologically, epithelial dysplasia and cellular atypia are prognostic indicators of premalignancy, which refers to impaired proliferation, maturation, and organization of the epithelium. These changes are seen in three degrees mild, moderate, and severe. Although the relationship between epithelial dysplasia and future carcinoma is not certain, it is generally stated that the degree of dysplasia and the transformation into cancer are directly proportional [6].

Technological advances in the last decade, especially with the advent of high-resolution digitized images and AI, have allowed pathology to adopt computational approaches, such as machine learning, to assess tissue aspects such as minimal or no human interference through algorithms capable of predicting, for example, precancerous lesions' risk of malignant transformation [7]. Thus, several studies have proposed using AI as a tool that adds to existing ones to understand the biology of these lesions better, but with the advantage of eliminating the pathologist's subjectivity regarding the interpretation of histopathological findings [8].

Considering the potential of this tool, this study investigated the nuclear aspects of OL and proliferative verrucous leukoplakia (PVL) cells with the main aim of detecting nuclear alterations and creating a classification algorithm that can be used for differential diagnosis between the two lesions. We hypothesized that the nuclear aspects investigated by AI are different between the two lesions and that this tool can be used for the purpose of differential diagnosis between an OL and PVL, especially in the early stages of both lesions when the clinicopathological aspects overlap, compromising the accuracy of the diagnosis both by the clinician but mainly by the pathologist.

The article "Segmentation of Oral Leukoplakia (OL) and Proliferative Verrucous Leukoplakia (PVL) Using Artificial Intelligence Techniques" was retracted in 2023. Reasons: signs of a paper mill; suspected computer-generated content; unreliable results or conclusions; lack of ethics approval or compliance.

## 2. Material and Methods

Sixty-one cases of OL, three cases of PVL, and five cases of SCC (all these cases were linked to malignant transformation of either OL or PVL) were collected from the Oral Pathology Laboratory of the Faculty of Dentistry of the University of Baghdad, Iraq, in the period from March 2021 to February 2022 to be used in the study in the neural network training, segmentation, and feature extraction phases. Initially, slides stained with hematoxylin and eosin used in the clinical routine were retrieved from their respective cases and reassessed to confirm the diagnosis of each of the lesions. In the case of OLs and PVLs, the degrees of dysplasia were also checked. For this diagnostic confirmation step, the criteria established by the World Health Organization of 2017 were used [9]. The fact of using routine slides stained with hematoxylin and eosin refers to the search in this work of the neural network to learn from the conditions found in oral pathology laboratories, ensuring better applicability of this tool. Clinicopathological data (lesion color, location, lesion type, dysplasia, malignant transformation, and size) and sociodemographic (gender, age, and smoking status) of the patients were obtained from the examination requests presented by the pathology laboratory. As a minimum inclusion criterion, only cases of OLs, PVLs, and SCCs had stained and well-preserved slides, and their respective diagnoses were used. Otherwise, the cases were excluded from the study.

### 2.1. Computer Analysis

The slides selected from each case were photographed using a Leica DM500 optical microscope to study the nuclei. On average, ten fields/lesions were obtained at 400× magnification, and all images were saved in JPEG and TIFF format with a resolution of 1600 × 1200. From the capture of these fields, the regions of interest were extracted. Then, the steps were used sequentially: segmentation, postprocessing, feature extraction, and classification, which are detailed below. All steps after extracting the ROIs were performed on a computer with the following configurations: AMD FX-8320 processor, 8GB of RAM, and NVIDIA GTX 1060 GPU with 6GB of VRAM. In the manual segmentation phase for network training, a Wacom Monitor-Cintiq was used to bypass the cores; the GIMP software was used both in this step and to obtain the ROIs obtained through the website https://www.gimp.org/. All software used in this work is available free of charge.

The article "Segmentation of Oral Leukoplakia (OL) and Proliferative Verrucous Leukoplakia (PVL) Using Artificial Intelligence Techniques" was retracted in 2023. Reasons: signs of a paper mill; suspected computer-generated content; unreliable results or conclusions; lack of ethics approval or compliance.

### 2.2. Segmentation

The first stage of segmentation is the training phase, in which the segmentation of the nuclei is performed manually from the ROIs extracted from the fields obtained from each lesion, as explained above. For this step, 481 ROIs were used, distributed as follows: 74 ROIs from OL without dysplasia, 77 ROIs from OL with mild dysplasia, 114 ROIs from OL with moderate dysplasia, 43 ROIs from OL with severe dysplasia, 59 PVL ROIs, and 114 SCC ROIs. A total of 15,027 cores were manually segmented and used in network training.

For training, the Mask R-CNN neural network was used together with the ResNet50 convolutional network to detect the cellular nuclei in the images. The ResNet50 convolutional network was first used in the learning stage of the characteristics of cell nuclei. The architecture of this network is shown in Figure 1. The network model is composed of 50 convolutional layers distributed over the input layer (E); four blocks of convolutional layers called Block 1 (B1), Block 2 (B2), Block 3 (B3), and Block 4 (B4); and an output step. Briefly, layer E has 64 convolutional filters with a size of 7 × 7 pixels that process the original image through a sliding window with an offset size of 2 pixels. Then, still in layer E, a max-pooling filter, with a size of 2 × 2 pixels, is used, with a displacement size equal to 2 pixels. This result is then applied to layer C1 of B1, which has 64 convolutional filters of size 1 × 1 pixel, followed by C2, which has 64 filters of size 3 × 3 pixels, and C3, which contains 256 filters of size 1 × 1 pixel. B1 is repeated three times over the image processed in layer E, totaling nine convolutional layers in this block. The result of B1 is applied to B2, passing first through layer C1, with 128 filters of size 1 × 1 pixel, followed by C2, with 128 filters of size 3 × 3 pixels, and C3, with 512 filters of size 1 × 1 pixel. This block has four repetitions, resulting in 12 convolutional layers. The result of B2 is then used in B3, which has 256 filters of size 1 × 1 pixel in C1, 256 filters of size 3 × 3 pixels in C2, and 1024 filters of size 1 × 1 pixel in C3. This block has six repetitions, totaling 18 layers. The result of B3 is used in B4, which also has three layers: C1, which has 512 filters of size 1 × 1 pixel, C2, with 512 filters of size 3 × 3 pixels, and C3, with 2048 filters of size 1 × 1 pixel. Block B4 is repeated three times, presenting nine layers in total. Finally, the generated data is transformed into a vector by an average pooling filter, while the softmax function is used to classify objects between core or background region. For this step, a fully connected layer with 1000 neurons is used. Between each block of convolutional layers (B1, B2, B3, and B4), the feature matrix is reduced in size by a proportionality of 2. For this, a sliding window with a displacement size of 2 pixels is used in the transition convolutions between each block. For the network model used in this work, the activation function adopted was the Rectified Linear Unit (ReLU) [10].

The article "Segmentation of Oral Leukoplakia (OL) and Proliferative Verrucous Leukoplakia (PVL) Using Artificial Intelligence Techniques" was retracted in 2023. Reasons: signs of a paper mill; suspected computer-generated content; unreliable results or conclusions; lack of ethics approval or compliance.

He and others [11] explained that the Mask R-CNN is a convolutional neural network that detects and separates candidate objects into distinct classes from regions. It consists of two stages; the first stage is called Region Proposal Network (RPN) and aims to generate sets of candidate objects in bounding boxes (the smallest square that comprises an object); the second stage aims to classify the objects contained in the bounding boxes and perform the regression of these boxes. In parallel to the second stage, the network also has a branch that provides a binary mask for each ROI.

This network detects and segments nuclei through the core characteristics extracted by ResNet50. For this, Mask R-CNN uses the feature maps generated by ResNet50 and stacks them from the largest (most detailed) to smallest (least detailed) map forming a Feature Pyramid Network (FPN). How ResNet50 has many layers that generate maps, the use of all of them can generate a large pyramid of high execution complexity. To get around this problem, only the last layer of each block is used, that is, C3 of the last B1, C3 of the last B2, C3 of the last B3, and C3 of the last B4. Then, the FPN layers are passed as input to the Region Proposal Network (RPN) to identify the cores in the top-down direction, from the smallest to the largest layer. With this, we classify the regions between core and background regions along with the bounding boxes in the first layer from above (smaller and less detailed). These results are then combined with the layers below, which are larger and have more detailed core features. As these results are passed through these larger, more detailed layers, the identified regions become more accurate and correct, while the bounding boxes are regressed. Finally, the R-CNN Mask through a convolutional network used in conjunction with feature maps produces a binary mask for each identified nucleus.

A multitasking loss rate is calculated for each region during the network training phase. This rate calculates the training error percentage, that is, how much the training is different from the gold standard (ROIs manually segmented by the expert). Basically, it sums the rate of loss (error) of classification and regression of boxes and masks, and its function is defined by

(1) $$\begin{array}{c} L=L_{\text{cls}}+L_{\text{box}}+L_{\text{mask}}. \end{array}$$

For the network model applied in this work, 60 ROIs were used for network training, 48 of them for training and 12 for testing, with 40 epochs performed in total.

416 ROIs were used to validate the model. Five of the total ROIs used were discarded during the process because they showed errors that prevented the program from working.

The article "Segmentation of Oral Leukoplakia (OL) and Proliferative Verrucous Leukoplakia (PVL) Using Artificial Intelligence Techniques" was retracted in 2023. Reasons: signs of a paper mill; suspected computer-generated content; unreliable results or conclusions; lack of ethics approval or compliance.

#### 2.2.1. Postprocessing

After the network classifies the objects between cores and the background region, some regions may be incompletely filled or even present noise or artifacts that can harm the segmentation process. To prevent this from happening, the postprocessing step is performed through morphological operations to eliminate false-positive regions and refine the segmented nuclei.

#### 2.2.2. Classification

The classification was performed using these vectors after the feature extraction process in which the *μ* and *σ* of the extracted nuclear features were transformed into a single vector for each ROI. The objective was to separate the images in the two different classes of lesions (OL and PVL) through the polynomial classifier (POL) [11]. This classifier employs polynomial expansion over the extracted feature vector to define the coefficients used in the separation of classes. For this to occur, the following discriminant polynomial function is used:

(2) $$\begin{array}{c} g\left(x\right)=a^{T}p_{n}\left(x\right). \end{array}$$

### 2.3. Statistical Analysis

To assess the method's effectiveness, a comparison was performed by estimating the overlap between the segmented images and the gold standard. With this, measures of true positives, false positives, true negatives, and false negatives are obtained, which were used in segmentation and classification. The ROC curve is obtained from the graph plotted by sensitivity versus false-positive rate (TFP). In order to compare the morphological characteristics of the nuclei between OLs and PVLs, regardless of the degree of dysplasia, the statistical Mann–Whitney tests or the unpaired *t*-test were used, according to the data distribution, as determined by the normality test, Shapiro-Wilk. It was considered statistically significant when *p* < 0.05.

## 3. Results

### 3.1. Clinicopathological Data

Most OL patients were male, while all PVL cases were female. The mean age of the patients was 55 years, 54 in the OLs and 72 in the PVLs. Most patients with OL were smokers, while only one patient with PVL had information about smoking. The main locations of both lesions were the buccal mucosa, tongue, alveolar ridge, and lip. For both OL and PVL, the most frequently found dysplastic alteration was mild dysplasia. Two cases of OL and one of PVL underwent a malignant transformation. Regarding the clinical characteristics of both lesions, most were white and had an average size of 1.5 cm.

The article "Segmentation of Oral Leukoplakia (OL) and Proliferative Verrucous Leukoplakia (PVL) Using Artificial Intelligence Techniques" was retracted in 2023. Reasons: signs of a paper mill; suspected computer-generated content; unreliable results or conclusions; lack of ethics approval or compliance.

#### 3.1.1. Nuclear Segmentation and Neural Network

For the analysis of nuclear segmentation of the lesions, photomicroscopy of the lesions of OL, PVL, and SCC was obtained, as described in the methodology. Of the total, 568 images of OL, 45 images of PVL, and 58 images of SCC were taken. From these images, the following numbers of ROIs were captured for each image: 1,217 ROIs from OL, 119 ROIs from PVL, and 133 ROIs from SCC. In this step, SCC samples were used to increase the number of nuclei used for neural network training purposes and increase its accuracy in the nuclear segmentation process. After obtaining the ROIs, the manual segmentation of the cellular nuclei belonging to the 481 ROIs selected for learning the algorithm was performed, which represented a supervised training phase. After that, the training of the Mask R-CNN network took place, where the network was fed with information about the cores in the training and the segmentation of cores by the network was performed in the separate ROIs for testing. To evaluate Mask R-CNN's performance in identifying and separating nuclei from background regions, both in testing and validation, the ROIs segmented by it were compared to the gold standard.

After training, Mask R-CNN was used to segment the ROIs extracted from the dataset, and the results of the segmentation process by Mask R-CNN can be seen in Figures 2–4.  Figure 2 shows the segmentation of an image with the nuclei being identified by the neural network. After training, it was found that the network successfully separated the nuclei from the background regions of the original image (Figure 2(a)). However, it was observed that the neural network detected perinuclear regions as belonging to the nuclear regions that were not identified in the gold standard (manual segmentation) and therefore were called false-positive nuclear regions (Figure 2(c), red arrow). This may be due to the similarity of coloration in the regions close to the nuclear limits. Still in Figure 2(c), it can be seen that the neural network did not identify some nuclear regions, as observed in the gold standard, indicating a false-negative result (green arrow). In addition, some segmented images presented noise that was wrongly classified as nuclei, which were considered false positives (Figure 2(e), red arrow). To correct these and other irregularities, a postprocessing step was carried out.

#### 3.1.2. Postprocessing

Postprocessing was carried out after segmentation by the neural network to correct some segmentation irregularities. The result can be seen in Figure 3. In this step, dilation (Figure 3(c)), hole filling (Figure 3(d)), and erosion (Figure 3(e)) operations were performed on an image. In Figure 3(b), the region indicated by the green arrow indicates the presence of a hole inside the core, where after the application of the expansion operation, the hole is reduced in size and, subsequently, eliminated by the hole-filling operation. At the end, the erosion operation was applied so that the nuclei returned to their respective original sizes. After the process of identifying the cellular nuclei, the tissues started to be classified based on the extraction of morphological characteristics from the objects classified as nuclei. The morphological characteristics studied were area (A), eccentricity (E), perimeter (PE), orientation (OR), solidity (S), entropy (EN), and Moran Index (IM). These selected characteristics are based on the work of which in turn was based on the studies [11, 12].

The article "Segmentation of Oral Leukoplakia (OL) and Proliferative Verrucous Leukoplakia (PVL) Using Artificial Intelligence Techniques" was retracted in 2023. Reasons: signs of a paper mill; suspected computer-generated content; unreliable results or conclusions; lack of ethics approval or compliance.

The area is calculated by the total value of the number of pixels in an object; eccentricity concerns the difference in the circumference of an object in relation to a circle, that is, the calculation of the elongation of objects; orientation calculates the relationship between the major axis of an object about the *x*-axis; solidity analyzes the deformity of an object, in the case of this work, the level of irregularity of the circular shape by the number of invaginations present.

The entropy measure analyses the intensity levels of a region and calculates the intensity variation present in the texture of a neighborhood of pixels. In this study, 7 neighborhood sizes were used to extract entropy measurements, as follows: 3 × 3, 5 × 5, 7 × 7, 9 × 9, 11 × 11, 13 × 13, and 15 × 15 pixels based on in the work of Kleppe et al. (2018). The Moran Index measures spatial autocorrelation by averaging the intensity of neighboring pixels and comparing them with the central pixel.

These 13 features were extracted for each core *n* present in all ROIs. In this way, each ROI has a matrix of size 13 × *n* and, from these matrices, the mean (*μ*) and standard deviation (*σ*) were extracted for each characteristic present in the ROI, generating two vectors (one for average and another for standard deviation), each having the descriptors of these characteristics: MK = [*m*_1_, *m*_2_ ⋯ *m*_13_] and DK = [*d*_1_, *d*_2_ ⋯ *d*_13_]. In MK, there is a vector with the average of all 13 features extracted from a given image, while in DK, there is a vector with the entire standard deviation of each feature found in the image in question. Finally, these vectors were concatenated (merged), forming a single vector that was used in the classification of each ROI.

The article "Segmentation of Oral Leukoplakia (OL) and Proliferative Verrucous Leukoplakia (PVL) Using Artificial Intelligence Techniques" was retracted in 2023. Reasons: signs of a paper mill; suspected computer-generated content; unreliable results or conclusions; lack of ethics approval or compliance.

The operation to eliminate small artifacts or noise classified as false positives was also performed.  Figure 4 shows the result of the operation that aims to eliminate segmented objects smaller than 30 pixels in an image, as identified by the red arrow in Figure 4(a).

The segmentation performed by the neural network obtained a satisfactory performance in identifying the nuclei and the background regions in the histological images, presenting an average accuracy of 92.95%.  Table 1 shows the means and standard deviations of sensitivity (SE), specificity (ES), accuracy (AC), correspondence rate (TC), and dice coefficient (DC) achieved by the Mask R-CNN network in segmenting the different tissue histopathological tests evaluated in this study. As can be seen, the values for each of the indices investigated in the neural network segmentation test were similar between the different lesions. In summary, these data indicate that the neural network presented similar sensitivity, specificity, and accuracy, indicating that the algorithm performed well in identifying cell nuclei in all cases.

### 3.2. Morphological Features Extracted by the Neural Network

The nuclear features extracted by the neural network were compared between OL and PVL. Altogether, the 13 characteristics used in the classification were extracted from the entire PVL ROI dataset and 1,196 of the 1,217 OL ROIs. Regarding entropies, seven entropy measures were used, and the data for each entropy/lesion can be seen in Table 2. The means for all entropies were always higher in the PVLs when compared to the OLs, and the differences were statistically significant (*p* < 0.0001).

The Moran Index revealed a statistically significant difference between OL and PVL, with means of 0.09702 and 0.1022, respectively (*p* = 0.0103). Regarding the area, the averages for OL and PVL were 836.4 and 1,050, respectively, with *p* < 0.0001. Similarly, the mean nuclear perimeters for OL and PVL were 103.3 and 117.9, respectively, with *p* < 0.0001. As for solidity, an average of 0.9685 and 0.9621 for OL and PVL was observed, respectively, with *p* < 0.0001. Regarding the eccentricity and orientation characteristics, the means for OL and PVL were very similar and with *p* > 0.05.

### 3.3. OL and PVL

For the separation between OL and PVL, a polynomial classifier was used. For this, 119 ROIs from PVL and 120 ROIs from OL randomly chosen were used by the classifier to assess the degree of separability between them. The classifier performed the cross-validation by dividing the ROIs into five groups (folds), where four of them were used for training and one for testing, which were alternated until all groups were trained and tested. As a result, the mean AUC of the classifier was 97.06%, the mean sensitivity was 95.83%, the mean specificity was 98.29%, and the mean accuracy was 97.05%. These results show that the classifier successfully distinguished the two lesions with a high degree of sensitivity, specificity, and accuracy, indicating that such a tool has great potential for use in the differential diagnosis between them. From the obtained results, it is possible to observe the results obtained in each group and the mean and standard deviation of the metrics used to evaluate the classifier's performance.

The article "Segmentation of Oral Leukoplakia (OL) and Proliferative Verrucous Leukoplakia (PVL) Using Artificial Intelligence Techniques" was retracted in 2023. Reasons: signs of a paper mill; suspected computer-generated content; unreliable results or conclusions; lack of ethics approval or compliance.

## 4. Discussion

This study aimed to investigate the detection of nuclear alterations in OLs and PVLs using a computer as well as the separation between them through the application of a classifier based on morphological nuclear characteristics. The results of this study shed light on one of the problems of oral pathology, which is to differentially diagnose a OL from a PVL, especially when the latter is at an early stage, which can generate inconsistencies, difficulties, doubts, and even diagnostic errors, according to pointed out by Al-Rawi (2022) [13]. Since our results showed the presence of detectable nuclear alterations among them, and that these alterations in turn were able to differentiate them with high precision by the polynomial classifier, this study showed the importance of investigating the cell nucleus through machine learning in DBPMs for diagnostic purposes as well as in the elucidation of the characteristic nuclear properties of each one of them. In light of advances in AI, this tool can be another foundation in the search for understanding these lesions together with studies aimed at finding differential molecular biomarkers between them, which do not exist to date.

Analyzing the clinicopathological data collected in this work, it can be seen that they are in line with the specific literature. In general, the incidence of OL was higher in males than in females; on the other hand, all cases of PVL were found in females, which are usually evidenced in studies involving these disorders [14]. Smoking, an important etiological factor of OLs, was also observed in most cases of OL investigated. As for the anatomical site, these lesions can develop anywhere in the oral cavity; however, the oral mucosa and the tongue are the regions constantly affected by them [15]. These aspects were also observed in our patients. Dysplasias, a histopathological finding commonly found in these lesions, were also present in most of our cases, mainly mild dysplasia and, more rarely, severe dysplasia. Although OL incidence is much higher than that of PVL, the rate of transformation of OLs is much lower. In our study, of the 61 cases of OL, only two underwent malignant transformation, while of the three cases of PVL, one patient only progressed to SCC, which in the light of our study can be considered high, even higher than the OLs used [14]. However, it is important to consider that our sample of PVL was small, which somewhat compromises the interpretation of this pathognomonic biological aspect of this lesion. In addition, there is the issue of the follow-up time of these patients, which seemed short to the point of detecting malignant transformation of their respective lesions, which led us to classify them as tumor-free in the present study. As for the color of the lesions, the vast majority of cases were white, a clinical aspect commonly found in these lesions, but which can alternate between white and red lesions in some cases [14, 15].

The article "Segmentation of Oral Leukoplakia (OL) and Proliferative Verrucous Leukoplakia (PVL) Using Artificial Intelligence Techniques" was retracted in 2023. Reasons: signs of a paper mill; suspected computer-generated content; unreliable results or conclusions; lack of ethics approval or compliance.

The model used in this study for learning and segmenting the cores was the Mask R-CNN network. The choice of this network came from the work of our study group in the area of AI carried out by, who used this network to identify nuclei in dysplastic lesions of the oral cavity developed in mice subjected to oral carcinogenesis by 4NQO. Mask R-CNN couples to ResNet50 or ResNet101 for learning the cores. We chose ResNet50 based on an empirical test carried out in the study by Silva (2019), which showed that ResNet50 performed better in targeting the dysplastic lesions investigated by him.

The different works on core identification have adopted different segmentation methods. In this regard, the Mask R-CNN proved to be the most effective in detecting nuclei in studies that compared different methods of nuclear identification. The study by Waal, Isaäc (2019) [16, 17], for example, segmented normal and abnormal nuclei of cervical cells using the Mask R-CNN, obtaining an average accuracy of 96%. They also compared this network with other segmentation methods and found that these methods presented lower results than the Mask R-CNN, such as the Multiscale Watershed + Binary Classifier, which achieved an accuracy of 88%, the RGVF of 83%, and Patch-based FCM of 85%. The work by Silva (2019) reached an average accuracy of 89.52% with the segmentation of nuclei of tongue epithelium cells without and with mild, moderate, and severe dysplasias. Also in this study, other methods were tested in comparison to his, and the results were inferior, such as the Otsu method, which presented an average accuracy of 60.78%, K-means of 77.32%, and SegNet of 73.12%. These data reveal that this neural network presents a good performance in terms of nuclear segmentation, which was confirmed by our accuracy results in OLs, PVLs, and SCCs, corresponding to 93.15%, 92.93%, and 94.63%, respectively. Future works may further improve this network so that its use in the area of pathology becomes ubiquitous, as shown by Anantharaman et al. (2018), who developed a network based on the Mask R-CNN exclusively for the detection of nuclei called Nuclei R-CNN, with even better results than the original Mask R-CNN.

The article "Segmentation of Oral Leukoplakia (OL) and Proliferative Verrucous Leukoplakia (PVL) Using Artificial Intelligence Techniques" was retracted in 2023. Reasons: signs of a paper mill; suspected computer-generated content; unreliable results or conclusions; lack of ethics approval or compliance.

As for the core features extracted from the entire OL and PVL dataset after neural network training, including entropy, Moran Index, area, perimeter, eccentricity, orientation, and solidity, they were compared between the two lesions. Significant differences were found between OL and PVL in the seven entropy levels evaluated in our study. Entropy is a measure that assesses the disorder of the nuclear texture, which, in turn, directly reflects the organization of chromatin and, consequently, the genetic and epigenetic changes that occur in the DNA molecule during the tumorigenesis process [18]. Thus, nuclear entropy has been studied in several types of cancers, focusing on determining clinical prognosis and tumor aggressiveness. In the study by, which investigated different types of cancers including the colon, ovary, uterus, prostate, and endometrium, it was observed that patients who exhibited more heterogeneous texture patterns, that is, higher entropy levels, had worse survival for all tumors evaluated. In our study, it is interesting to note that all mean entropy levels analyzed were higher in PVLs than in OLs, suggesting a greater chromatin disorder in those lesions to the detriment of these, which partly may explain the greater potential of PVLs to progress to SCC.

Similarly, [19] found a consecutive increase in entropy in the epithelial cell nuclei of nonsmoking smokers and patients with precancerous conditions. Therefore, these entropy results seem to be useful in distinguishing lesions with lower and higher malignant transformation potential, in the case of LB and PVL, respectively, suggesting the occurrence of distinct genetic and epigenetic alterations between them. Further studies will assess whether higher entropy indices in OLs indicate a greater risk of malignant transformation, as seems to be the case for PVLs.

Another characteristic evaluated in our study and related to the nuclear texture is the Moran Index. There are no works in the literature that use the Moran Index to assess cell nuclei, except for Silva (2019). As in our study, in work by Silva (2019), this feature proved useful in distinguishing the different lesions studied, with significant differences between healthy tissue and tissue with dysplasia; in the present work, a significance was obtained between OL and PVL. In this sense, it can be concluded that both entropy and the Moran Index can be used to detect changes in chromatin in premalignant lesions, a fact reinforced by the study by [20–22], who analyzed some nuclear characteristics and verified that the nuclear texture is an effective variable in differentiating the degrees of dysplasia in Barrett's ssophagus, in addition to being efficient in predicting progression to cancer, which, together with our results, further highlights the importance of evaluating the nuclear textures in an attempt to elucidate the pathological conditions of premalignant lesions.

The article "Segmentation of Oral Leukoplakia (OL) and Proliferative Verrucous Leukoplakia (PVL) Using Artificial Intelligence Techniques" was retracted in 2023. Reasons: signs of a paper mill; suspected computer-generated content; unreliable results or conclusions; lack of ethics approval or compliance.

Regarding the area, our results point to a direct relationship with some studies on DBPMs. The work of [23] showed that the area of the cellular nuclei of the oral submucosal fibrosis lesion with dysplasia was greater than that of the normal nuclei, suggesting that this alteration could indicate the occurrence of tumorigenesis, reflecting the increase in the metabolic activity of these cells. Similar to the area, perimeter reflects the size of nuclei and is sometimes used together with area to infer changes in nuclear size. The work by Krishnan et al. (2010) showed an increase in the perimeter of the nuclei between oral submucosal fibrosis with dysplasia and normal oral mucosa. Solidity is a descriptor used in the assessment of nuclear deformity. In our results, a significant difference was found between the two injuries, also proving to be a useful variable in distinguishing between OL and PVL. Here, the mean solidity in the PVLs was slightly lower than in the OLs. Unlike our study, work by Krishnan et al. [23] found no significant differences in the solidity of nuclei in an attempt to discriminate oral submucosal fibrosis from normal oral mucosa. Similarly, the study [19] also did not detect substantial differences in nuclear solidity between nonsmoking smokers and patients with PMBD. One hypothesis is that PVLs have a high power of malignant transformation compared to other MPDs, increasing the chances of nuclear deformity and leaving the nuclei less convex and more irregular, a characteristic found in cancer cells, as described. Solidity is a variable that is still little investigated in studies involving the evaluation of nuclear morphology by computational algorithms. Therefore, it is expected that further research may include it in the evaluation of nuclei in different DBPMs as a possible descriptor that characterizes different lesions, as observed in our study.

The article "Segmentation of Oral Leukoplakia (OL) and Proliferative Verrucous Leukoplakia (PVL) Using Artificial Intelligence Techniques" was retracted in 2023. Reasons: signs of a paper mill; suspected computer-generated content; unreliable results or conclusions; lack of ethics approval or compliance.

We found no significant differences in eccentricity and orientation between OL and PVL. Interestingly, the study by [24–28] also found no differences in eccentricity between oral submucosal fibrosis nuclei and buccal mucosa. Thus, further studies should be conducted in order to determine the value of these variables in DBPMs more clearly. Thus, it is possible to conclude from our investigation that both lesions carry distinct nuclear alterations. Our findings also support the importance of the nuclear study from computational techniques evaluated by an AI, a promising area in medicine that, without a doubt, will shape the field of pathology soon, finding new ways to interpret the pathological processes that occur. In various diseases. Based on the evidence found in our study and in the works mentioned here, these descriptors may prove to be useful in predicting the progression to SCC of PMBDs, such as OL and PVL. The investigated nuclear features were transformed into vectors so that the classifier could dichotomize the samples between the two lesions. The classifier used all 119 PVL ROIs and 120 OL ROIs to assess the degree of separability. It is worth mentioning that for the classification to perform well, it is important to have a balanced number among the samples to be investigated. Therefore, only 120 OL ROIs were used by the classifier [29–33].

The polynomial classifier proved to be very effective in the studies in which it was adopted, with extremely satisfactory performance [15] in the classification between normal and abnormal tissues of mammograms through texture analysis, reaching an AUC of 98%, a performance superior to the SVM, decision tree, and K-NN classifiers, which were also compared in the study. Similarly, in work by Silva (2019), the polynomial classifier achieved an average AUC of 92% in the classification between healthy tissues and those with different degrees of dysplasia, that is, a superior result than the multilayer perceptron, decision tree, and random classifiers. Forest was compared in their study. Similarly, our result was excellent, with an average UAC of 97.06%, indicating that this classifier can be an additional tool for pathologists in defining a histopathological diagnosis since the diagnosis of PVLs is still a constant challenge in oral pathology, and that can be easily confused with OLs, especially in the initial cases. Thus, our study proposes the use of AI as a tool that raises the criteria currently adopted in the distinction between these two lesions, reducing the margin of doubt and improving the accuracy of the diagnosis with less subjectivity. Further studies are needed to verify whether this method can be used in the early stages of PVLs, when they are usually labeled as OLs without any evidence of evolution to more aggressive forms, which would be of great importance in determining an early diagnosis of PVLs, increasing the chances of successful treatment.

The article "Segmentation of Oral Leukoplakia (OL) and Proliferative Verrucous Leukoplakia (PVL) Using Artificial Intelligence Techniques" was retracted in 2023. Reasons: signs of a paper mill; suspected computer-generated content; unreliable results or conclusions; lack of ethics approval or compliance.

## 5. Conclusion

Based on the investigations carried out in this work, the present study showed that, despite being histologically similar, OLs and PVLs carry distinct nuclear properties that can be used for differential diagnosis between them, thus, helping to resolve one of the major challenges of oral pathology in the search for more effective and accurate ways to establish the differential diagnosis between OL and PVL. The fact that the neural network has achieved an excellent performance in nuclear identification through the supervised training performed reveals that this method can be a great ally in our later works involving histological studies, including the analysis of more cases of OLs and PVLs in the first time. In addition, the characteristics found in the nuclei of the two lesions can provide important information in the construction of a model to assess the risk of malignant transformation of these disorders, being extremely important in making therapeutic decisions for each case. Added to this, the use of a classifier could also be used in the future as an additional tool for cases of a difficult diagnosis. Finally, our investigations are added to the various works that show machine learning as a new possibility for studies in pathology, being an effective, low-cost method that will possibly be used on a large scale in the near future in clinical routines, adding speed, precision, and prediction in diagnoses.

## Figures and Tables

**Figure 1:** Architecture of the ResNet50 neural network used in the segmentation process for the learning of cell nuclei.

**Figure 2:** Segmentation of an OL image by the gold standard and the neural network. (a) Original image; (b) mask resulting from the gold standard; (c) mask resulting from the Mask R-CNN neural network showing false-positive (red arrow) and false-negative (green arrow) regions; (d) segmentation resulting from (c) and image of SCC showing a small noise that was classified as false positive (red arrow); (e) mask resulting from Mask R-CNN; (f) segmentation resulting from (a).

**Figure 3:** Postprocessing step in a SCC image: (a) original image, (b) mask after segmentation, (c) mask after the dilation operation, (d) mask after applying the hole-filling operation, (e) mask after erosion operation, and (f) resulting segmentation.

**Figure 4:** Operation to eliminate small artifacts in an SCC image: (a) resulting mask of the neural network; (b) segmentation resulting from (a); (c) mask resulting from the process of eliminating objects smaller than 30 pixels; (d) segmentation resulting from (c).

The article "Segmentation of Oral Leukoplakia (OL) and Proliferative Verrucous Leukoplakia (PVL) Using Artificial Intelligence Techniques" was retracted in 2023. Reasons: signs of a paper mill; suspected computer-generated content; unreliable results or conclusions; lack of ethics approval or compliance.

**Table 1:** Result of the segmentation of the Mask R-CNN in the different histopathological tissues of OL, PVL, and SCC.

Lesion	SE (%)	ES (%)	AC (%)	TC (%)	DC (%)
OL	81.89 ± 6.44	96.51 ± 2.28	93.15 ± 2.76	74.95 ± 8.21	83.80 ± 5.60
PVL	80.79 ± 4.58	96.64 ± 1.61	92.93 ± 2.34	74.77 ± 5.71	83.82 ± 3.90
SCC	80.24 ± 9.28	97.67 ± 1.83	94.63 ± 2.85	74.42 ± 8.81	83.47 ± 6.36

**Table 2:** Values of the seven levels of nuclear entropy evaluated between OL and PVL.

Variable	Measures of central tendency and dispersion	LB	LVP	*p*-value
Entropy 3 × 3	Average	1968	2137	<0.0001∗
	Median	1983	2149	
	Minimum	1428	1962	
	Maximum	2314	2284	

Entropy 5 × 5	Average	2769	3049	<0.0001∗
	Median	2784	3082	
	Minimum	2017	2759	
	Maximum	3308	3268	

Entropy 7 × 7	Average	3243	3598	< 0.0001∗
	Median	3252	3.64	
	Minimum	2363	3232	
	Maximum	3913	3862	

Entropy 9 × 9	Average	3566	3974	< 0.0001∗
	Median	3571	4024	
	Minimum	2587	3552	
	Maximum	4.33	4266	

Entropy 11 × 11	Average	3804	4249	< 0.0001∗
	Median	3805	4308	
	Minimum	2735	3785	
	Maximum	4636	4574	

Entropy 13 × 13	Average	3986	4459	< 0.0001∗
	Median	3987	4518	
	Minimum	2836	3962	
	Maximum	4872	4811	

Entropy 15 × 15	Average	4.13	4624	< 0.0001∗
	Median	4.13	4687	
	Minimum	2909	4101	
	Maximum	5059	5	

∗Mann–Whitney test; ∗∗unpaired *t*-test.

## Data Availability

The data used to support the findings of this study are included within the article.
